The article "Evaluating the Clinical Outcomes of Remdesivir Among Patients Admitted With COVID-19 in a Tertiary Care Hospital" was retracted in 2022. Reasons: false authorship; lack of ethics approval or compliance; concerns about the data; concerns about the authorship.

# Evaluating the Clinical Outcomes of Remdesivir Among Patients Admitted With COVID-19 in a Tertiary Care Hospital

**DOI:** 10.7759/cureus.19487

**Published:** 2021-11-11

**Authors:** Ahmad G Butt, Jahanzeb Ahmed, Syed Muhammad Huzaifa Shah, Camilo Andrés Avendaño Capriles, Hady Al-Rihani, Bilal Ahmed, Muhammad Salman, Arti Devi, Sher Wali

**Affiliations:** 1 Biology, University of Western Ontario, London, CAN; 2 Internal Medicine, Shalamar Institute of Health Sciences, Lahore, PAK; 3 Medicine, Ziauddin University, Karachi, PAK; 4 Clinical Research, Harvard Medical School, Boston, USA; 5 Medicine, Universidad del Norte, Barranquilla, COL; 6 Surgery, Rafik Hariri University Hospital, Beirut, LBN; 7 Internal Medicine, Central Park Medical College, Lahore, PAK; 8 Epidemiology and Public Health, Indus Hospital & Health Network, Karachi, PAK

**Keywords:** sar-cov 2 infection, impact, treatment, clinical outcomes, covid-19, remdesivir

## Abstract

Introduction: This study was conducted to determine whether remdesivir administration for treatment of coronavirus disease 2019 (COVID-19) is associated with reducing deaths among COVID-19 hospitalized patients.

Methodology: It was a retrospective study, and the data was acquired at Ziauddin Hospital in Karachi, Pakistan. All patients admitted between February and May 2021 with severe acute respiratory syndrome coronavirus 2 (SARS-Cov-2) infection confirmed by polymerase chain reaction testing from nasopharyngeal samples were included in the study, including those who received at least five-day treatment of remdesivir and who did not receive even a single dose of remdesivir.

Results: Data of overall 174 patients were used, out of which 71 (40.80%) received remdesivir. After propensity score matching, 71 patients in the remdesivir group were successfully matched with the non-remdesivir patients on the basis of age, gender, and disease severity. Results of multivariable logistic regression showed that there is no significant difference in deaths between patients who received remdesivir and patients who did not receive remdesivir (p-value=0.122). However, the length of hospital stay was significantly lower in the remdesivir group than in the control group (p-value=0.001).

Conclusion: Results of this study can provide evidence that remdesivir can be efficient in reducing the duration of COVID-19 illness, and a five-day course of treatment is sufficient for patients to get clinical benefits.

## Introduction

As of February 2, 2021, the pandemic caused by the severe acute respiratory syndrome coronavirus 2 (SARS-CoV-2) was still going strong, with more than 103 million cases and more than two million deaths occurring all over the world [1]. Even though vaccines have played a significant contribution in reducing disease burden and its seriousness but they are not 100% effective in preventing the disease [2]. Studies have been done to assess the effectiveness of various pharmacological agents for the treatment of coronavirus caused by SARS-CoV-2 [3]. One of the drugs is remdesivir that has achieved a lot of attention. It is a nucleotide analog prodrug that has been proved to be efficient against different RNA viruses [4]. Researchers around the world have come up with conflicting results regarding the effectiveness of remdesivir [5]. On the basis of Adaptive coronavirus disease 2019 (COVID-19) Treatment Trial (ACTT-1) results, the FDA in the United States approved remdesivir for the treatment of COVID-19 infected hospitalized patients [6]. On the other hand, WHO did not approve remdesivir use on the basis of the Solidarity trial [7].

Even though the findings of the Solidarity trial suggest that remdesivir does not have a significant mortality benefit for COVID-19 patients alone, however, remdesivir still may play a significant role in shortening the duration of disease and reducing the severity of illness, both of which are important outcomes when hospitals are overburdened with COVID-19 patients [8]. Receiving remdesivir was linked to a considerably shorter time to clinical improvement in the retrospective multicenter research [9]. The remdesivir group had a decreased mortality rate, but the difference was not statistically significant. The review conducted by Ansems et al. found that remdesivir makes little or no difference to all-cause mortality among patients with COVID-19. Additionally, remdesivir may have no or little effect on the duration to liberation from invasive mechanical ventilation. However, insufficient data were available to determine the impact of remdesivir on mortality across different subgroups [10].

Considering the number of admissions because of Covid-19 in Pakistan, remdesivir can be effective in shortening admission time, especially in a country like Pakistan, where lack of healthcare resources is one of the big issues. However, not enough studies have been done in this region regarding the effectiveness of this drug on the length of ICU stay. Therefore, this study has been conducted to determine whether remdesivir administration for treatment of COVID-19 is associated with reducing deaths or the length of hospital/ICU stay among COVID-19 hospitalized patients.

## Materials and methods

It was a retrospective study comprised of the data gathered from Ziauddin Hospital, Karachi, Pakistan. The study was reviewed by the Ethics Review Committee of Ziauddin Hospital (2021-01-005) and was determined exempt from ongoing IRB review.

All patients admitted with SARS-Cov-2 infection confirmed by polymerase chain reaction (>30 ct) testing from nasopharyngeal samples between February 2021 to May 2021 were included in the study including those who received at least five-day treatment of remdesivir and who did not receive even a single dose of remdesivir. Patients who were discharged against medical advice and those who were pregnant were excluded from the analysis. Lastly, patients in which remdesivir treatment was stopped due to any reason were also not included in the final analysis as the study assessed five-day remdesivir course efficacy. Besides this, patients who were discharged within 24-hours of hospital stay were also excluded.

The healthcare organization's remdesivir policy follows the guidelines from the FDA. The organization prescribed remdesivir to patients who were prescribed with remdesivir, have required to have a significant illness (extracorporeal membrane oxygenation or mechanical ventilation or oxygen saturation <94% requiring supplemental oxygen or breathing ambient air), and whose alanine aminotransferase level was less than five times the upper reference limit.

The primary outcome was either patient was discharged alive from the hospital with significant clinical improvement reported in the patient’s file or death. Secondary outcomes were the number of days of patient admission in hospital from the first remdesivir treatment day. All the data were gathered from the hospital management information system (HMIS) or patient’s file. Data including the age of the patient at the time of admission, gender of the patient, smoking status, vital signs at the time of admission, laboratory tests on the day of admission, the severity of disease (computed using Charlson comorbidity index), and comorbidities were extracted from HMIS.

Statistical analysis

Data analysis was done using STATA Statistical Software. Release 16 (StataCorp. 2019. College Station, TX: StataCorp LLC). Logistic regression was used to estimate the association between remdesivir treatment and outcome. Demographic characteristics, laboratory results, and clinical variables were included in the analysis based on clinical knowledge and interest. We used propensity score matching using gender, age, and disease severity to create pairs of individuals, with one patient treated and the other patient being the most similar patient eligible, to account for nonrandomized remdesivir assignments and different timing of initial administration. Propensity scores were calculated from the logistic regression model using receiving remdesivir as the outcome. Analysis was done on the matched data sets taking (discharge alive vs. death) as outcome using multivariable logistic regression. A p-value less than 0.05 was considered significant.

## Results

Of the 260 patients admitted to the Ziauddin Hospital with COVID-19 between February 2021 and May 2021, 90 patients were excluded from the analysis. The reasons for their exclusion were patients did not complete five-day treatment of remdesivir (n=40) due to any reason, discharge from hospital within 24 hours (n=21), leave against medical advice (n=12), death within 24 hours (n=9) of admission, and others (n=9). Among the remaining 174 patients, 71 (40.80%) received remdesivir. Of those patients receiving remdesivir, the mean age was 55.49 years (±13.49); 11 (15.49%) were women). After propensity score matching, 71 patients in the remdesivir group were successfully matched with the non-remdesivir patients on the basis of age, gender, and disease severity. Table 1 shows the demographic and clinical characteristics of remdesivir recipients and controls before propensity score matching, and Table 2 shows the demographic and clinical characteristics of remdesivir recipients and controls after propensity score matching.

**Table 1:** Characteristics of Patients Before Propensity Score Matching *Mean (Standard Deviation)

Variable	Control n(%)	Remdesivir n(%)	Absolute standardized difference
Age*	51.46 (16.94)	55.49 (13.49)	0.26
Gender			
Male	80 (77.67)	60 (84.51)	0.17
Female	23 (22.33)	11 (15.49)	
Smoking Status			
Non-smoker	87 (84.47)	54 (76.06)	0.21
Current Smoker	16 (15.53)	17 (23.94)	
Vital Signs*			
Systolic BP (mmHg)	136.10 (26.46)	139 (15.28)	0.13
Diastolic BP (mmHg)	78.97 (16.79)	78.88 (12.67)	0.005
Pulse (beats/min)	104.8 (25.33)	105.7 (19.38)	0.04
SpO2	88.46 (12.35)	80.04 (14.21)	0.63
Respiratory Rate (breathe/min)	30.33 (10.15)	33.35 (9.61)	0.31
Laboratory Results*			
Hemoglobin, g/dL	12.28 (3.15)	13.12 (1.71)	0.33
Platelet count, ×103 /μL	279.1 (197.36)	261.9 (101.41)	0.11
White blood cell count, cells/μL	23.32 (75.12)	14.87 (14.21)	0.15
Absolute lymphocyte count, /μL	13.72 (10.10)	10.77 (5.29)	0.36
Past Diagnosis			
Diabetes	41 (39.81)	28 (39.44)	0.01
Hypertension	38 (36.89)	30 (42.25)	0.11
Chronic kidney disease	9 (8.74)	1 (1.41)	0.33
COPD or chronic lung disease	4 (3.88)	2 (2.82)	0.06
Disease Severity			
Mild	14 (13.59)	4 (5.63)	0.08
Moderate	40 (38.83)	10 (14.08)	0.55
Severity	23 (22.33)	19 (29.76)	0.05
Critical	26 (25.24)	38 (53.52)	0.26

**Table 2:** Characteristics of Patients After Propensity Score Matching *Mean (Standard Deviation)

Variable	Control n(%)	Remdesivir n(%)	Absolute standardized difference
Age*	54.25 (16.70)	55.49 (13.49)	0.08
Gender			
Male	60 (84.51)	60 (84.51)	0.00
Female	11 (15.49)	11 (15.49)	
Smoking Status			
Non-smoker	61 (85.92)	54 (76.06)	0.25
Current Smoker	10 (14.08)	17 (23.94)	
Vital Signs*			
Systolic BP (mmHg)	139.10 (27.06)	139.00 (15.28)	0.01
Diastolic BP (mmHg)	80.48 (16.92)	78.88 (12.67)	0.11
Pulse (beats/min)	105.40 (29.79)	105.70 (19.37)	0.01
SpO2	86.56 (13.18)	80.04 (14.21)	0.47
Respiratory Rate (breathe/min)	31.74 (11.03)	33.35 (9.61)	0.15
Laboratory Results*			
Hemoglobin, g/dL	12.50 (3.01)	13.12 (1.71)	0.25
Platelet count, ×103 /μL	309.60 (207.33)	261.90 (101.41)	0.29
White blood cell count, cells/μL			
Absolute lymphocyte count, /μL	13.07 (11.02)	10.77 (5.29)	0.26
Past Diagnosis			
Diabetes	35 (49.30)	28 (39.44)	0.20
Hypertension	29 (40.85)	30 (42.25)	0.02
Chronic kidney disease	9 (12.68)	1 (1.41)	0.44
COPD or chronic lung disease	3 (4.23)	2 (2.82)	0.07
Disease Severity			
Mild	7 (9.86)	4 (5.63)	0.06
Moderate	16 (22.54)	10 (14.08)	0.03
Severity	23 (32.39)	19 (26.76)	0.04
Critical	25 (35.21)	33 (53.52)	0.11

Results of multivariable logistic regression showed that there is no significant difference in clinical outcome between patients who received remdesivir and patients who did not receive remdesivir (p-value=0.122), as shown in Table 3 after adjusting for all other confounding variables. Another variable significantly associated with clinical outcome was the severity of disease (p-value<0.05). The odds of death are 2.61 and 2.71 times more in patients with critical and severe disease, respectively, than patients with mild disease.

**Table 3:** Multivariable Logistic Regression on Effect of Treatment on Outcome * Significant at p-value<0.05 AOR: Adjusted odds ratio

Variable	AOR (95% CI)	p-value
Group		
Remdisivir	0.68 (0.33, 1.39)	0.137
Non-Remdisvir		
Disease Severity*		
Mild		
Moderate	0.78 (0.17, 3.47)	0.328
Severity	2.61 (1.47, 5.05)	0.005
Critical	2.71 (1.49, 5.02)	0.002

Of the 140 matched individuals (70 remdesivir and 70 matched controls), 37 (51.39%) patients who received remdesivir and 35 (48.61%) patients who did not receive remdesivir were discharged alive from hospital after significant clinical improvement, with a mean time of discharge of 12.13 (±4.23) days for remdesivir recipients and 14.88 (±2.87) days for controls. There is a significant difference in length of stay between the remdesivir and control group (p-value=0.001).

## Discussion

A global priority is to optimize the use of medicines to reduce COVID-19 associated mortality and morbidity. Remdesivir has been the topic of debate because the ACTT-1 research, funded by the National Institutes of Health, indicated a shorter time to positive clinical outcomes. However, the bigger Solidarity study, funded by WHO, found no effect in terms of mortality. Even though the findings of the Solidarity trial showed that remdesivir does not show any significant impact on the mortality rate among serious COVID-19 patients, but it can play an important role in decreasing the severity of illness and duration of illness. This is important for lower- and middle-income countries that are overwhelmed with COVID-19 patients [8]. It can reduce the burden on hospitals. In the current study, the mortality rate was lower in the remdesivir group as compared to the non-remdesivir group, but the difference was not statistically significant. The magnitude of this association was similar to the ACCT-1 study [6]. However, the current study has found that length of stay and in-hospital was shorter in the remdesivir group than in the non-remdesivir group. The retrospective study conducted by Garibaldi et al. in 2021 also found that patients who received remdesivir had a significantly shorter time to clinical improvement [9].

We included only those patients who received at least five days of remdesivir that supported the recommendations for an initial five-day course for most patients. In the ACTT-1 study, a 10-day treatment course of remdesivir was used, and a five-day and 10-day comparison showed similar efficacy [11]. In another study to assess the efficacy of a five-day course treatment course of remdesivir, it has been shown that a 5-day course was significantly associated with improvement in disease severity [12]. Findings of our study that show that a 5-day course of treatment is associated with clinical benefits are vital, especially considering the situation of availability of remdesivir in Pakistan and hospitals where it can provide greater benefits.

Considering the preliminary results from different clinical trials about remdesivir, the FDA authorized the use of the drug in May 2020 for treatment in children and adults hospitalized with COVID-19. Since then, remdesivir has received conditional or full approval in certain countries. However, considering that no impact of remdesivir on mortality rate has been seen in the current study and in past studies, it is evident that remdesivir alone is not sufficient for patients. Therefore, to continue to improve outcomes in patients with Covid-19, a number of therapeutic methods, including novel antivirals, immune response modifiers, and combination therapies, are needed.

The current study has certain limitations; therefore, the findings of this study should be interpreted with caution. First, it was a retrospective study; thus, the number of important variables were not assessed, such as time of death and concomitant medications. Second, the sample size is very small, and data were used from one tertiary care hospital. Therefore, the generalizability of this is low. In the future, prospective studies need to be conducted in different centers and assess the efficacy of different drugs with remdesivir that can reduce mortality rate and create a positive impact on clinical outcomes in patients with severe Covid-19. 

## Conclusions

The current study suggested that remdesivir is associated with a significant reduction in the hospital stay among patients admitted to hospitals for treatment of COVID-19. Results of this study can provide evidence that remdesivir can be efficient in reducing the duration of COVID-19 illness, and a five-day course of treatment is sufficient for patients to get clinical benefits.
